# The Effect of Crank Length Changes from Cycling Rehabilitation on Muscle Behaviors

**DOI:** 10.1155/2021/8873426

**Published:** 2021-04-26

**Authors:** Lu Zongxing, You Shengxian, Wei Xiangwen, Chen Xiaohui, Jia Chao

**Affiliations:** School of Mechanical Engineering and Automation, Fuzhou University, No. 2 Xueyuan Road, Fuzhou, 350116 Fujian, China

## Abstract

**Background:**

Many sports and physical activities can result in lower limb injures. Pedaling is an effective exercise for lower extremity rehabilitation, but incorrect technique may cause further damage. To some extent, previous experiments have been susceptible to bias in the sample recruited for the study. Alternatively, methods used to simulation activities can enable parametric studies without the influence of noise. In addition, models can facilitate the study of all muscles in the absence of the effects of fatigue. This study investigated the effects of crank length on muscle behavior during pedaling.

**Methods:**

Six muscles (soleus, tibialis anterior, vastus medialis, vastus lateralis, gastrocnemius, and rectus femoris), divided into three groups (ankle muscle group, knee muscle group, and biarticular muscle group), were examined under three cycling crank lengths (100 mm, 125 mm, and 150 mm) in the present study. In addition, the relationship between crank length and muscle biological force was analyzed with the AnyBody Modeling System™, a human simulation modeling software based on the Hill-type model. *Findings*. Based on inverse kinematic analysis, the results indicate that muscle activity and muscle force decrease in varying degrees with increases in crank length. The maximum and minimum muscular forces were attained in the tibialis anterior and vastus lateralis, respectively. *Interpretation*. Studying the relationship between muscle and joint behavior with crank length can help rehabilitation and treating joint disorders. This study provides the pedal length distribution areas for patients in the early stages of rehabilitation.

## 1. Introduction

Nowadays, cycling plays an important role in people's daily life and rehabilitation. However, lower limb injuries often occur during cycling. Injuries of the lower limb, including the hip, knee, and ankle can occur if pedaling parameters (e.g., crank length) are not set appropriately or due to overuse. There are three classifications for lower limb injuries, under overuse and common cycling [1–3].

First, cyclists may develop hip problems, such as trochanteric bursitis, which is due to the repetitive sliding of the fascia lata over the greater trochanter. This can result from a high seat position. Furthermore, high-seat can also cause trochanteric synovitis and iliopsoas tendinitis. Second, knee joint injuries are the most common injures from cycling. Knee injuries account for 62% of all overuse injuries, and many cyclists suffer from lateral, anterior, and medial knee pain. Of there, lateral knee pain is the most common knee joint injury. The overuse of bicycles is considered the main reason for these injuries. The third class of injuries encompasses ankle and foot problems. When riding long distances, it is very common to sustain a foot injury. Cycling in low seating positions with a high pedaling frequency can cause ankle and foot injuries, and an incorrect pedal position under the foot may cause metatarsalgia.

Pedaling exercise has been widely used in the rehabilitation of lower limb injuries [4]. Rehabilitation with cycling involves interactions between the nervous system, bones, and muscles. Understanding the relationship between body structures and cycling parameters (such as seat height and crank length) is not only important for patients to perform rehabilitative exercises but can also guide healthy people to perform physical activities safely. For example, setting an appropriate crank length [5–7], pedaling cadence [8], and the pedal condition [9, 10] (pedal height and pedal position) affects the outcomes of rehabilitation. Martin and Spirduso [8] divided 710 feasible pedal places into 16 groups for modeling and simulation and found that knee joint forces were smaller near saddle position (SP). Conversely, the ankle and hip joints in the far SP per saddle height (SH) were minimal. Therefore, understanding changes in muscle strength and reaction forces when pedaling provides insights that can be used to guide rehabilitation.

Many previous studies [11–13] have used electromyography (EMG) to examine the activation patterns of lower limb muscles during pedaling.

In contrast, this study has used the AMS (AnyBody Modeling System™) for simulation pedaling with different crank lengths. The AMS software transforms parts of the human body, which is a very complex structure [14], into rigid body systems for analysis [15]. In this study, a Hill-type [16] biomechanical model of cycling exercise (AnyBody software version 6.0, AnyBody Technology, Aalborg, Denmark) was used involving 84 muscles in the lower extremities based on the criteria for muscle recruitment [17, 18].

There are several limitations of research on multibody dynamics, such as the verification and validation of musculoskeletal models and simulations. For studies on musculoskeletal modeling, Rasmussen and colleagues [19, 20] used dynamics and anatomical knowledge to continually modify and refine the model, so that the Hill-type musculoskeletal model better conformed to actual human movements. In the process of verifying the model, it was difficult to obtain EMG signals in vivo. Previous studies [21, 22] investigated muscle behavior during cycling, observing acceptable agreement in the changes in muscle activation based on contrasting analyses with other models.

The effect of cycling crank length on muscle behaviors requires parametric further investigation. Both experimental and simulation methods can be used to study the factors that influence muscle behavior during cycling. While human experiments are susceptible to sample bias, simulation studies allow the examination of complex body systems by changing only one parameter in the absence of noise from other confounding variables [23]. In addition, models can facilitate the study of all muscles in the absence of fatigue [24, 25]. As much, models provide valuable insight into biomechanical variables that are difficult to measure directly (for example, muscle force and joint reaction force) and offer improvements upon many previous studies addressing joint kinetics [26] and cycling cadence [27] that can be directly measured.

The purpose of this study was to reveal the relationship between muscle activity and muscle force with different crank lengths during the pedaling rehabilitation. The outcomes may help to provide physicians with objective guidance for programming bicycling for rehabilitation.

## 2. Methods

The AMS is a human simulation software that provides human musculoskeletal models. The model used in this study had 84 muscles in the lower limb, incorporating three degrees of freedom at the hip (flexion/extension, abduction/adduction, and internal/external rotation), one degree of freedom at the knee (lateral movement along the *y*-axis), and two degrees of freedom at the ankle (flexion/extension and abduction/adduction). In the AMS, all body segments are modeled as rigid bodies to eliminate the influence of soft tissues and other uncertainties.

In the process of establishing the model, the first step was to determine the position of the world coordinate system, which was set to [0, 0, 0] (the red coordinate system in Figure 1). The center of the pedal coincided with the world coordinate system. At the same time, the angle of the knee and ankle were adjusted to represent actual human cycling. After these adjustments, the joint angles of both the knee and the hip were 90 degrees. In addition, to ensure the accuracy of the experiment, it was necessary to determine variables other than the crank length that should remain unchanged. After a series of adjustments, the final parameters were as follows: the seat position was [-0.7, 0.55, 0]; the contact point between the foot and the pedal was set to [*L*, 0, 0.15] (right crank point), [-L,0, -0.15] (left crank point). “*L*” represents the crank length. In the model, there were five segments in total, each of which had six degrees of freedom. The human body model had a total of 30 degrees of freedom. Six constraints were added to the pelvis and seat through the stdjoint, while the hip, knee, and ankle had three, five, and four constraints, respectively. There are one constraint of the knee joint (lateral movement along the *y*-axis) and two constraints of the ankle joint (flexion/extension and abduction/adduction). Three constraints were added between the foot and the pedal by using a spherical joint. Finally, the remaining degrees of freedom was determined by the driving function of the pedal. In total, there were 29 constraints. If a mechanism is needed to perform a certain movement, the number of its original moving parts should be equal to the number of degrees of freedom. In the model, the original actuator was only a pedal rotation, and since there was one degrees of freedom in the mechanism, the model met the conditions for movement to occur.

In this study, 25 torque loads were added to the pedal. Since the pedal driver had no motor, the torque had to be balanced by the muscles in the system. After the model was established, the relevant biomechanical parameters were analyzed by modifying crank length. A preliminary determination of three crank lengths was conducted at 100 mm, 125 mm, and 150 mm. Every time the crank length changed, a kinematic analysis was performed again to verify the feasibility of the model. Then, an inverse kinematic analysis was conducted to obtain the data. Figure 1 shows an overview of the model analysis process. All whole lower limb muscles were divided into three groups: the knee muscle group (vastus medialis (VM) and vastus lateralis (VL)), the ankle muscle group (soleus (SOL) and tibialis anterior (TA)), and the biarticular muscle group (gastrocnemius (GAS) and rectus femoris (RF)). Several of the most representative muscles were selected for further analysis. The musculotendon parameters were set using constant values from the patient-specific musculoskeletal model (Table 1).

In the AMS, careful consideration must be given to muscle recruitment. Muscle recruitment refers to the overall efficiency of muscle use. The solution for muscle recruitment in inverse dynamics is usually expressed as a mathematical optimization problem. The goal is to minimize the value by the objective function *G*(*f*^(*M*)^).

(1) $$\begin{array}{c} G\left(f^{\left(M\right)}\right)=\overset{n^{\left(M\right)}}{\underset{i=1}{\sum }}{\left(\frac{f_{i}^{\left(M\right)}}{N_{i}}\right)}^{p}. \end{array}$$

Subject to

(2) $$\begin{array}{c} {Cf}^{\left(M\right)}=d, \end{array}$$

(3) $$\begin{array}{c} 0\leq f^{\left(M\right)}\leq N_{i},\;i\in \left(1,2\cdots n\right), \end{array}$$

where *G* is the objective function of the mathematical optimization problem, and its solution depends on the maximum of the unknown force in the problem. In Equation (1), *F*_*i*_ and *N*_*i*_ represent muscle force and muscle strength, respectively. The *i* is the *i*th muscle, and the power of the polynomial criterion (*p*) in the AMS shows the synergy between the muscles. To ensure the minimum value of fatigue strength, *p* = 3 [30]. Redundancy in the muscle system can be expressed by equilibrium Equation (2), where *C* is the coefficient matrix, and *d* is the vector used to represent all known forces. Equation (3) indicates the nonnegativity constraint on muscle forces. This means that within a certain strength range (0-*N*_*i*_), the muscle can only be pulled but not pushed. Moreover, in the AMS, all muscles have a preset strength; exceeding this muscle strength will cause further injury, and the system will also report errors, which must be avoided in modeling.

In the AMS, the position of the *i*th body is described by Equation (4), where *r*_*i*_ is the global position vector of the center of mass and *p*_*i*_ is the vector of four Euler parameters.

(4) $$\begin{array}{c} q_{i}={\left[r_{i}^{T}q_{i}^{T}\right]}^{T}. \end{array}$$

When modeling, taking the right leg as an example, the crank angle changes as shown in Figure 2, and the angle changes can be plotted as shown in the figure.

The crank drive equation determines the movement of the foot pedal and is described as follows:

(5) $$\begin{array}{c} \varphi =\overset{3}{\underset{i=1}{\sum }}\left[A_{i}\cos\left(w_{i}t\right)+B_{i}\sin\left(w_{i}t\right)\right], \end{array}$$

(6) $$\begin{array}{c} w_{i}=\left(i-1\right)2\pi f, \end{array}$$

(7) $$\begin{array}{c} B=\left[B_{1},B_{2},B_{3}\right], \end{array}$$

where *φ* is the pedal angle. *A*_*i*_ and *B*_*i*_ are the Fourier coefficients, and *ƒ* is the natural frequency; *w*_*i*_ is the angular frequency (*w*_2_ is equivalent to the angular velocity of the crank). The components of *A* and *B* control foot motion during cycling.

The crank torque pattern by means of a sine function was described as follows:

(8) $$\begin{array}{c} M=M_{\text{offset}}+\left(M_{\text{offset}}-M_{\text{TDC}}\right)\sin\;\left(4\pi f+\alpha_{M}\right). \end{array}$$

In Equation (8), the crank torque *M*_TDC_ at the top of the pedal cycle and the phase angle *α*_*M*_ at the top of the pedal cycle are independent variables and were determined during the optimization process. *M*_offset_ represents the input data. The angular frequency of the torque function was twice the frequency of the circular pedal frequency, due to the inclusion of two legs in the model [21].

## 3. Results

The changes in muscle activity during pedaling with a 100 mm crank length can be seen in Figure 3. Activation of the ankle muscle group (SOL and TA) was sensitive from 0° to 135°, showing an initial increase followed by a decrease in the activity. The SOL reached its maximum activity at 45°, but the TA reached its maximum at 90°. Moreover, the knee muscle group (VL and VM) was active at the beginning and end of the motion, with the activity of the VL and VM muscles first increasing and then decreasing. The activity of the VL and VM reached peak muscle at 265°. The peak muscle activity of the VL was the largest of all muscles. The GAS muscle was active from 0° to 225°. The activity of the GAS was relatively weak in the 225° to 360° range. The RF muscle was active throughout the cycle, reaching peak muscle activity at 200°.

The activity of the TA, VL, and RF muscles when pedaling under three different crank lengths have is shown in Figure 4. The trend in muscle activity was roughly the same under different crank lengths. The time points at which the peak occurs and activity begins are roughly the same, and this also shows the accuracy of the established model to some extent. As crank length increases, muscle activity decreases.

Figure 5 shows the variation in the muscular force of six muscles under three different crank lengths. As the crank length increased, muscle force decreased. The peak muscle force of the TA was the smallest, being only 166 N. The change in muscle force was not accompanied by a measurable change in crank length. Peak muscle force was reduced from 166 N in the 100 mm condition to 110 N in the 150 mm condition. While the peak force of the VL was the largest of all muscles, up to 1321 N, the decrease in muscle force was also the greatest, as peak force decreased from 1321 N in the 100 mm condition to 859 N in the 150 mm condition, a reduction of 462 N. The SOL and VM muscles only participated in the motion between 0°--45° and 225°--360°. Variation in SOL muscle force at different crank lengths was relatively weak, while variation in the VM force at different crank lengths was larger than that of the SOL. The force of the TA was very small throughout the whole pedaling cycle, only generating force in the middle and early stages of the cycle. The force of the GAS was only active in the 0°--225° range, peaking at 50° with 689 N. The force of the RF changed in the initial and final stages, but in the second half, the trend was more obvious.

In Figure 6, the maximum muscle force of each muscle at different crank lengths is shown. The change in the maximum muscle force of each muscle can be clearly seen. Among these muscles, the maximum muscle force was in the VL and the lowest was from the TA. With increases in crank length, all maximum muscle forces were decreased.

## 4. Discussion

Pedaling is enabled by a coordinated sequence of leg muscle contractions, of which the SOL, TA, VL, VM, GAS, and RF muscles all make an important contribution. A wide variety of methods have been used to study the biomechanics of pedaling. In one study, the inertial load on the crank was set to 150 W and 250 W [31], and a different range of cycling (such as 9 kg/m^2^ to 36 kg/m^2^ and 56 kg/m^2^ to 182 kg/m^2^) was used to study pedaling modeling. Some studies have used different saddle positions with 182 feasible pedaling places [4]. Setting an appropriate crank length is an important issue. In some studies [32–34], kinematic and inverse kinematic analyses have been used to investigate the behaviors of cycling power output and cadence with different crank lengths. However, all these previous studies have focused on *t* external forces, not biological forces. In this study, the effect of three crank lengths (100 mm, 125 mm, and 150 mm) on muscle kinetics (muscle activity) and muscular force was investigated.

The previous studies investigated the relationship between crank length and muscle behavior. For example, Macdermid and Edwards [7] investigated seven female cross-country mountain bike athletes to examine the effect of different crank lengths (170 mm, 172.5 mm, and 175 mm) on power output during cycle ergometry at a constant cadence (50 rpm). In this paper, only the relationship between crank length and power output was studied.

According to Hicks' research [35], the validation of a model requires multiple steps. One important limitation is the lack of verification of in vivo EMG signals on the premise of missing comparative data. Alternatively, validation can be achieved by comparing the model and simulation data to independent experiments and other models. In order to prevent secondary injury during rehabilitation, it is necessary to avoid muscle activation greater than its maximum capacity. The maximum activity of the VL muscle was higher than all other muscles. The maximum activity of the TA muscle was the lowest of all the muscles. This study showed that the SOL muscle was active from the top to the bottom of the pedal cycle and that the VL muscle was inactive during the middle stage of pedaling.

In the ankle muscle group, the active phases of the SOL and TA muscles were staggered, such that the SOL muscle was active during the 0°–45° and 230°–360° sections of the pedaling cycle, while the TA muscle was active between 45° and 225° of the cycle. Comparing the force curves of the two muscles, the TA produced a smaller force than the SOL. In the ankle muscle group, the SOL provided the most muscle force during the pedaling cycle. In the knee muscle group, the activity of the VL and VM muscles was basically the same through the whole cycle, but the muscle force of the VL was larger than that of the VM. The active stages of the GAS and RF muscles were also different, as the GAS was active during 0°–225°, while the RF was active during 180°–360° of the cycle.

## 5. Conclusion

Among the six muscles, maximum peak muscular force and peak muscle activity were achieved by the VL muscle, while the minimum peak muscular force and peak muscle activity were identified in the TA muscle.

Muscle activity and force generation were reduced with increases in crank length. The VL had the largest variation, and the TA had the smallest variation.

In the rehabilitation process, these findings could determine a more appropriate treatment plan according to the changes in muscle force and muscle activity.

Crank length is only one of the factors determining muscle activation and force generation. Other factors may also have an impact on pedaling, and environmental parameters must be adjusted according to the actual situation.

## Figures and Tables

**Figure 1:** Analysis process of the influence of crank length on muscle behavior during cycling.

**Figure 2:** Variation in crank angles during movement.

**Figure 3:** The activity of each muscle when the crank length was 100 mm.

**Figure 4:** The activity of the TA, VL, and RF muscles during a cycle (0°-360°) with different crank lengths (100 mm, 125 mm, and 150 mm). (a) TA, (b) VL, and (c) RF.

**Figure 5:** The muscle force of six muscles during a cycle (0-360°) in the different crank lengths: (a) SOL, (b) TA, (c) VL, (d) VM, (e) GAS, and (f) RF.

**Figure 6:** Maximum muscle force of each muscle in different crank lengths.

**Table 1:** Musculotendon parameters, based on and adapted from Ward et al. [28] and Millard et al. [29].

Muscle segment	Optimal force (N)	Optimal fiber length (cm)	Tendon slack length (cm)	Pennation angle (°)
Soleus (SOL)	6195	4.4	27.7	21.9
Tibialis anterior (TA)	1227	6.8	24.1	11.2
Vastus medialis (VM)	2748	9.7	20.0	24.2
Vastus lateralis (VL)	5149	9.9	22.1	14.5
Gastrocnemius (GAS)	1575	5.9	37.6	12.0
Rectus femoris (RF)	2192	7.6	44.9	12.4

## Data Availability

We confirm the data are available from the first author or corresponding author on reasonable request.
